The article "Measurement and Impactors of Tourism Carbon Dioxide Emission Efficiency in China" was published in 2022. Journal: J Environ Public Health.

# Measurement and Impactors of Tourism Carbon Dioxide Emission Efficiency in China

**DOI:** 10.1155/2022/9161845

**Published:** 2022-07-14

**Authors:** Guohua Jiang, Anding Zhu, Jun Li

**Affiliations:** ^1^School of Tourism and Culinary Arts, Zhejiang Business College, Hangzhou 310053, China; ^2^School of Management and E-Business, Zhejiang Gongshang University, Hangzhou 310018, China; ^3^School of Digital Economy & Trade, Wenzhou Polytechnic, Wenzhou 325035, China

## Abstract

With tourism carbon dioxide emission efficiency (TCDEE) as an undesired output, this study establishes an index system based on the inputs and outputs of TCDEE and measures the provincial TCDEE of China in 2010–2018, using the epsilon-based measure (EBM). In addition, the impactors of TCDEE were tested by the Tobit model. The main results are as follows: China's TCDEEs had obvious provincial differences. Only six provinces reached the efficient frontier of TCDEE, namely, Beijing, Tianjin, Inner Mongolia, Shanghai, Jiangsu, and Guangdong. The other provinces failed to reach this state, leaving a room for improvement. Most eastern provinces had relatively high TCDEEs, while the central and western provinces had relatively low TCDEEs. In the sample period, the TCDEEs in eastern, central, and western parts all changed in the shape of letter N. The TCDEEs of the eastern part were much higher than those of the central and western parts. According to the results of the Tobit model, TCDEE is clearly enhanced by the urbanization level, strongly inhibited by industrial structure, technical progress, opening-up, and environmental regulation, and not significantly affected by the tourism level.

## 1. Introduction

Global warming, a result of the greenhouse effect, brings an unprecedented challenge to our survival and development. China pays much attention to this problem and takes multiple measures to reduce the emissions of carbon dioxide, such as environmental governance, energy saving, and green, low-carbon technology. Every sector in China attaches great importance to reducing carbon dioxide emissions.

Tourism, a pillar industry of the national economy, is energy-intensive [1]. From the angle of carbon dioxide emissions, traveling is a healthy but high-carbon lifestyle. The carbon dioxide emitted by tourism has become a major inducer of environmental degradation. Statistics show that tourism contributes about 5% of carbon dioxide emitted around the world [2]. In recent years, tourism has developed rapidly at an annual rate of 10% in China. Despite its economic benefits, the extensive growth model of tourism consumes lots of energy and emits more and more carbon dioxide year by year. Therefore, the efficiency and sustainable development of regional tourism hinge on the increase of tourism carbon dioxide emission efficiency (TCDEE).

To date, very few scholars have fully evaluated the low-carbon tourism economy in China [3]. A few researchers have explored the carbon dioxide emission of tourism [4, 5] but failed to fully understand the TCDEE in each province. Besides, very few scholars have discussed which factors that greatly affect the TCDEE. To fill up the gap, this paper scientifically evaluates the TCDEE in each province of China and further explores the influencing factors of this efficiency. The research findings help to fully understand the development level of low-carbon economy in tourism and facilitate the formulation of proper carbon reduction policies.

## 2. Literature Review

The estimation of tourism carbon dioxide emission has long attracted the attention of the academia. Early on, some scholars recognized that the carbon dioxide emitted by tourism is a major driver of global warming. For example, Scott et al. [6] regarded tourism as one of the main industries emitting greenhouse gases. Peterson and Dubois [7] found that the greenhouse gases generated by tourism are responsible for 4.4% of global warming, and the percentage grows by 3.2% each year in 2005–2035.

Many scholars strive to estimate the carbon dioxide emitted by tourism by scientific methods. Currently, tourism carbon dioxide emissions can be measured by two approaches. The first approach is top-down analysis. Taking tourism as a part of national economy, the top-down analysis estimates the carbon dioxide emitted by tourism by the input-output method and social accounting matrix method. Through top-down analysis, Perch-Nielsen et al. [8] estimated the carbon dioxide emitted by domestic tourism of Switzerland as 6.62 Mt. Berners-Lee et al. [9] combined the input-output method and lifecycle process analysis to estimate the greenhouse gas emissions of northwestern England.

The second approach is the bottom-up analysis, which divides the tourism participants into tourists and tourism enterprises. This approach estimates the carbon dioxide emitted by tourism, using lifecycle process analysis, sampling survey, and carbon footprints. For example, Gössling et al. [10] estimated tourism carbon dioxide emissions from three aspects: transportation, lodging, and tourism activities. Mayor and Tol [11] forecasted the trend of tourism carbon dioxide emissions through scenario analysis, according to index data such as tourist conditions, tourism energy consumption, and tourism income.

TCDEE is an important indicator of the relationship between the development of tourism economy and the carbon dioxide emitted by tourism. The effective measurement of TCDEE provides an important reference for determining the energy-saving and emission reduction level of regional tourism. The existing studies mainly concentrate on the efficiencies of tourism hotels [12, 13], travel agencies [14, 15], and tourism transportation [16, 17]. Some scholars discussed the ecological efficiency of tourism under environmental constraints [18, 19].

Because of the difficulty in estimating the TCDEE, the above estimations of TCDEE mainly focus on the national scale. The research on the scale of province, municipality directly under the central government, and autonomous region (hereinafter collectively referred to as the province) is severely lacking. What is worse, the literature on TCDEE mainly focuses on an aspect of tourism, such as tourism hotel and tourism transport. There is little in the report that discusses the carbon efficiency of the entire tourism industry. In addition, none of the above studies recognizes the benefit of taking TCDEE as an undesired output: reflecting the constraint of environmental factors on tourism development and facilitating the accurate evaluation of the low-carbon development level of tourism.

To fill up the research gap, this study adopts the bottom-up method to estimate tourism carbon dioxide emission and builds an index system for TCDEE containing an undesired output. In addition, the epsilon-based measure (EBM) was adopted to estimate the TCDEE of each province in China, and the TCDEE impactors were verified using the Tobit model.

## 3. Methodology

### 3.1. EBM Model

Data envelopment analysis (DEA) is more adaptable and flexible than stochastic frontier analysis (SFA) because it can handle problems with many inputs and outputs, without needing a production function. In view of this, our research adopts DEA to measure TCDEEs in China.

The earliest DEA models have constant or variable returns to scale [20, 21]. The DEA model with constant returns to scale assumes that the returns to scale of inputs remain unchanged. However, this assumption goes against the reality, resulting in wrong efficiency measurement. Some scholars improved the DEA model with constant returns to scale into a DEA model with variable returns to scale. But the improved model still seeks the maximal output, failing to consider undesired outputs, which are inevitable in actual production. Hence, the improved model may seriously under/overestimate the efficiency. In addition, the above traditional DEA models ignore nonradial slack variables [22].

To overcome the defects of traditional radial DEA models, Tone [23] proposed the slack-based measure (SBM) model, which soon gained common recognition in the academia. The greatest advantage of the model is the consideration of both undesired outputs and nonradial slack variables. As a result, the efficiency estimated by SBM is close to the actual situation of the production process. Nevertheless, SBM has several shortcomings in efficiency measurement. Firstly, the measured efficiency tends to be smaller than the actual level, for the model overlooks the proportion between the input and output targets and the actual values. The underestimation of efficiency increases the slackness of inputs and outputs, calling for significant changes to inputs and outputs for efficiency improvement. Secondly, the optimal slackness of zero values differs significantly from that of positive values, which further amplifies the error in efficiency measurement.

Tone and Tsutsui [24] extended the SBM into the EBM model, drawing on the merits of the DEA model with constant returns to scale. This hybrid model supports both radial and nonradial inputs and outputs, providing a new way to evaluate the efficiency of decision-makers. The main ideas of EBM are as follows:

In a complete production system, there are *n* decision-makers responsible for making decisions about production. The *k*-th decision-maker is denoted by DMU_*k*_=(*x*_*k*_, *y*_*k*_, *b*_*k*_). The system can produce *p* desired outputs *y* and *q* undesired outputs *b*, after receiving *r* inputs *x*. For clarity, the inputs, desired outputs, and undesired outputs are denoted by *X*=(*x*_1_, *x*_2_,…, *x*_*n*_) ∈ *R*_+_^*r*×*n*^, *Y*=(*y*_1_, *y*_2_,…, *y*_*n*_) ∈ *R*_+_^*p*×*n*^, and *B*=(*b*_1_, *b*_2_,…, *b*_*n*_) ∈ *R*_+_^*q*×*n*^ vectors. Thus, all possible production scenarios can be expressed as *T*={(*x*, *y*, *b*) : *x* can produce *y* and *b*}. Then, the EBM model can be established as:

(1) $$\begin{array}{c} \theta^{*}=\min\frac{\phi -\sigma_{x}\sum_{i=1}^{r}w_{i}^{-}s_{i}^{-}/x_{ik}}{\rho +\sigma_{y}\sum_{o=1}^{p}\left(w_{o}^{+}s_{o}^{+}/y_{ok}\right)+\sigma_{b}\sum_{u=1}^{q}\left(w_{u}^{b-}s_{u}^{b-}/b_{uk}\right)},\\ s_{.}t_{.}\phi x_{ik}=\sum_{t=1}^{n}x_{it}\lambda_{t}+s_{i}^{-},\;i=1,\ldots ,r,\\ \rho y_{ok}=\sum_{t=1}^{n}y_{ot}\lambda_{t}-s_{o}^{+},o=1,\ldots ,p,\\ \rho b_{uk}=\sum_{t=1}^{n}b_{ut}\lambda_{t}+s_{u}^{b-},u=1,\ldots ,q,\\ \lambda >0,\;s_{i}^{-},s_{o}^{+},s_{u}^{b-}\geq 0, \end{array}$$

where 0 < *θ*^*∗*^ ≤ 1 is the TCDEE; *s*_._*t*_._ is the model constraint; *x, y,* and *b* are the input, desired output, and undesired output, respectively; *r*, *p,* and *q* are the total number of inputs, desired outputs, and undesired outputs, respectively; *i*, *o,* and *u* are corresponding to an input or an output; *ϕ* is the programming parameter for the radial part of the model; *σ*_*x*_ is the core parameter containing both the radial effect *ϕ* and nonradial effect *s*_*i*_^−^; *σ*_*y*_ and *σ*_*b*_ are the core parameters containing nonradial effects *s*_*o*_^+^ and *s*_*u*_^*b*−^, respectively; *ρ* is the nonradial programming parameter of the model; *x*_*ik*_, *y*_*ok*_, and *b*_*uk*_ are the *i*-th input, oth desired output, and *u*-th undesired output of DMU_*k*_, respectively; *w*_*i*_^−^, *w*_*o*_^+^, and *w*_*u*_^*b*−^ are the weights of the *i*-th input, oth desired output, and *u*-th undesired output, respectively; *s*_*i*_^−^, *s*_*o*_^+^, and *s*_*u*_^*b*−^ are the slack terms of the *i*-th input, oth desired output, and *u*-th undesired output, respectively; *t* and *λ* are the decision-maker and it weight, respectively. *x*_*rt*_, *y*_*ot*_, and *b*_*ut*_ are the input, desired output, and undesired output of *t* DMUs; *k* is the efficiency of the *k*-th DMU to be estimated.

If *s*_*i*_^−^, *s*_*o*_^+^, and *s*_*u*_^*b*−^ are not zero, then *θ*^*∗*^ is smaller than 1. In this case, the decision-maker fails to achieve the optimal efficiency and needs to improve the inputs and outputs. If and only if *s*_*i*_^−^ =  *s*_*o*_^+^ =  *s*_*u*_^*b*−^ = 0, the decision-maker achieves the efficiency of 1, reaching the efficient frontier. In this case, there is no need to improve inputs and outputs.

### 3.2. Index System

As a total factor, TCDEE refers to the maximum tourism output and minimum carbon dioxide emissions from constant inputs such as capital, labor, and energy. Referring to Zha et al. [25], this study builds up an index system of TCDEE based on relevant inputs and outputs. Notably, the desired outputs include the total tourism income and total number of tourists, while the undesired output is tourism carbon dioxide emissions. The definition of each index is given in Table 1.

#### 3.2.1. Labor

Many sectors, such as industry and agriculture, provide tangible products. Meanwhile, tourism provides intangible products called services. The services are provided by the employees of scenic areas, restaurants, travel agencies, etc. In general, the labor input can be best characterized by the number of tourism employees and their effective labor time. However, the effective labor time of tourism employees is not available in relevant statistical yearbooks. This study decides to measure the labor input by the number of tourism employees.

#### 3.2.2. Capital

In addition to labor, capital is an essential input of tourism development. Specifically, the fixed assets in tourism not only promote infrastructure construction but also improve the services of scenic areas, thereby enhancing tourism quality and attractiveness. Considering data availability, this study takes the original value of the fixed assets in tourism in each province as the capital index. To eliminate the effect of price-induced inflation, the nominal fixed assets in tourism were deflated to the actual fixed assets in tourism with 2005 as the base year, using the fixed asset price index.

#### 3.2.3. Energy

The tourism energy consumption is not provided in relevant statistical yearbooks. Thus, this study estimates the consumption with the tourism consumption stripping coefficient. Three sectors are closely associated with tourism, namely, transportation, warehousing, and postal industry; wholesale and retail industry; lodging and catering industry. The energy consumed in these sectors is partially related to tourism and must be stripped out by the right ratio. The tourism energy consumption can be estimated by

(2) $$\begin{array}{c} E_{it}=\sum_{pq}E_{pq\cdot t}\cdot \alpha_{q}\cdot R_{it}, \end{array}$$

where *E*_*it*_ is the tourism energy consumption of the *i*-th province in the *t*-th year; *E*_*pq*·*t*_ is the terminal consumption of the *q*-th energy in the *p*-th sector in the *t*-th year; *α*_*q*_ is the coefficient of 10,000 tons of standard coal for the *q*-th energy; and *R*_*it*_ is the tourism consumption stripping coefficient of the *i*-th province in the *t*-th year.

#### 3.2.4. Desired Outputs

The desired outputs reflect the yield of tourism development. Total tourism income and the total number of tourists are the two most important indicators of regional tourism development. Both were selected as desired outputs.

Total tourism income refers to the total operating income of tourism enterprises by providing tourists with tourism products and services. This index directly measures the economic value created by tourism development and sets a standard for measuring the scale of regional tourism. To eliminate the effect of price-induced inflation, the nominal total tourism income was deflated into the actual total tourism income with 2010 as the base year, using the consumer price index.

The total number of tourists reflects the attractiveness of regional tourism, as well as the service quality and development scale of tourism in a region. Therefore, it is very suitable to take this index as a desired output. For convenience, this study substitutes the total number of tourists with the number of inbound overnight tourists in each province.

#### 3.2.5. Undesired Output

The carbon dioxide emitted by tourism is not directly given in relevant statistical yearbooks. Drawing on the results of Becken et al. [26], Becken, and Patterson [27], this study employs the bottom-up method to estimate the tourism carbon dioxide emissions, which mainly come from three tourism-related sectors: tourism transportation, tourism lodging, and tourism activities. Thus, the carbon dioxide emitted by tourism can be estimated by

(3) $$\begin{array}{c} C=C_{T}+C_{H}+C_{R}, \end{array}$$

where *C* is the total carbon dioxide emitted by tourism; *C*_*T*_, *C*_*H*_, and *C*_*R*_ are the carbon dioxide emitted by tourism transportation, tourism lodging, and tourism activities, respectively.

(4) $$\begin{array}{c} C_{T}=\sum_{i=1}^{n}N_{ti}\cdot g_{i}\cdot \lambda_{i}, \end{array}$$

where *n* is one of the four transportation modes, namely, railway, highway, waterway, and civil aviation; *N*_*ti*_ is the passenger turnover of the *i*-th transportation mode in the *t*-th year; *g*_*i*_ is the proportion of the *i*-th transportation mode in passenger turnover; and *λ*_*i*_ is the carbon dioxide emission factor of the *i*-th transportation mode.

(5) $$\begin{array}{c} C_{H}=\sum 365\cdot R_{i}\cdot Q_{i}\cdot \beta , \end{array}$$

where *R*_*i*_ and *Q*_*i*_ are the mean occupancy rate and number of beds of starred hotels in the *i*-th province, respectively; *β* is the carbon dioxide emission factor per bed per night of starred hotels in the *i*-th province [28].

(6) $$\begin{array}{c} C_{R}=\sum_{h=1}^{n}Z\cdot Y_{h}\cdot \delta_{h}, \end{array}$$

where *h* is one of the five tourism activities, namely, sightseeing, vacation, business trip, visiting relatives/friends, and others; *Z* is the number of tourists; *Y*_*h*_ and *δ*_*h*_ are the tourist composition and carbon dioxide emission factor of the *h*-th tourism activity, respectively.

After sorting out the relevant literature, the carbon dioxide emission factors of railway, highway, waterway, and civil aviation were set to 72 gCO_2_/pkm, 133 gCO_2_/pkm, 106 gCO_2_/pkm, and 137 gCO_2_/pkm, respectively; the carbon dioxide emission factor per bed per night of starred hotels in the *i*-th province was set to 2.458 gCO_2_/p visitor-night; the carbon dioxide emission factors of sightseeing, vacation, business trip, visiting relatives/friends, and others were set to 417 gCO_2_/p visitor, 1,670 gCO_2_/p visitor, 786 gCO_2_/p visitor, 591 gCO_2_/p visitor, and 172 gCO_2_/p visitor, respectively.

### 3.3. Tobit Model

This study focuses on the impactors of TCDEE. Referring to Sun et al. [29], and considering data availability, the authors decided to explore how six factors, out of the various external impactors of tourism carbon emissions, affect TCDEE, namely, tourism level (TL), industrial structure (IS), technical progress (TP), opening-up (OU), urbanization level (UL), and environmental regulation (ES).

#### 3.3.1. Tourism Level (TL)

Tourism level is closely related to regional eco-environment. On the one hand, the level of tourism directly manifests the economic benefits of that industry. On the other hand, the improvement of the regional tourism level leads to better tourism infrastructure and tourism services, which benefit the increase of TCDEE. Referring to Qiu et al. [30], this study measures the tourism level with per capita tourism income. The natural logarithm of the variable was added to the model.

#### 3.3.2. Industrial Structure (IS)

The industrial structure reflects the proportion of primary, secondary, and tertiary industries in the national economy. The energy consumption and pollution emissions of tourism depend closely on the development of tertiary industries, namely, transportation, warehousing, and postal industry; wholesale and retail industry; lodging and catering industry. Hence, this study characterizes the industrial structure with the proportion of the tertiary industry in the gross domestic product (GDP) and thereby analyzes the relationship between the industrial structure and tourism carbon dioxide emissions.

#### 3.3.3. Technical Progress (TP)

Technical progress has a major impact on energy-saving, emission reduction, and environmental efficiency of a region. The introduction of new techniques, processes, and products to regional tourism enterprises helps to lower the energy consumption of regional tourism and promotes the sustainable growth of tourism. Considering data availability, this study represents technical progress by the ratio of regional expenditure on research and development (R&D) to GDP.

#### 3.3.4. Opening-Up (OU)

As China further opens to the world, more and more tourists are attracted to this country. The growth of inbound tourists stimulates the demand for tourism services and pushes up the emissions of carbon dioxide. Meanwhile, opening-up makes it easier for China to import cutting-edge technology of environmental governance and advanced experience of tourism management. These technology and experience promote energy conservation and emission reduction in tourism and thus improve TCDEE. Overall, the influence of opening-up over TCDEE remains uncertain and is yet to be verified. This study converts USD into RMB by the mean exchange rate and characterizes opening-up with the ratio of actual foreign direct investment (FDI) utilized in each province to GDP.

#### 3.3.5. Urbanization Level (UL)

The rising level of urbanization improves the infrastructure in towns and cities and promotes the quality of the service industry, laying a solid basis for tourism development. The urbanization process also encourages the aggregation of talents and industries, which favors the carbon dioxide reduction of tourism. This study substitutes the urbanization level with the proportion of permanent urban residents in total regional population.

#### 3.3.6. Environmental Regulation (ES)

Tourism, as an energy-intensive industry, inevitably emits a huge sum of carbon dioxide in its development. The government plays an important role in carbon reduction of tourism. By investing more in environmental pollution control, the government forces tourism enterprises to control pollutant discharge and reduce carbon dioxide emissions. If the investment is too high, however, the resource allocation mechanism of the market would be distorted, leading to the green paradox [31]. Considering data availability, this study characterizes environmental regulation with the proportion of the investment on environmental pollution control in GDP.

Through the above analysis, this study sets up a regression model for TCDEE impactors. As the explained variable, TCDEE ranges between 0 and 1. If the ordinary least squares (OLS) method is adopted to estimate TCDEE, the estimation would be biased, for the value range of the TCDEE violates the OLS assumption that the value of explained variable is unlimited. To solve the problem, Tobin [32] designed the Tobit model to handle censored explained variables. Hence, this study establishes a Tobit model for TCDEE impactors, which explains TCDEE from the angles of the tourism level, industrial structure, technical progress, opening-up, urbanization level, and environmental regulation

(7) $$\begin{array}{c} {\text{TCEE}}_{it}^{*}=\alpha +\beta_{1}{\text{TL}}_{it}+\beta_{2}{\text{IS}}_{it}+\beta_{3}{\text{TP}}_{it}+\beta_{4}{\text{OU}}_{it}+\beta_{5}{\text{UL}}_{it}+\beta_{6}{\text{ES}}_{it}+\varepsilon ,\\ \left\{\begin{array}{c} {\text{TCEE}}_{it}={\text{TCEE}}_{it}^{*}\left(\text{if }{\text{TCEE}}_{it}^{*}<1\right),\\ {\text{TCEE}}_{it}=1\left(\text{if }{\text{TCEE}}_{it}^{*}\geq 1\right), \end{array}\right. \end{array}$$

where TCEE is the explained variable of TCDEE; TL, IS, TP, OU, UL, and ES are the tourism level, industrial structure, technical progress, opening-up, urbanization level, and environmental regulation, respectively (Table 2); *β*_1_, *β*_2_, *β*_3_, *β*_4_, *β*_5_, and *β*_6_ are the coefficients of the tourism level, industrial structure, technical progress, opening-up, urbanization level, and environmental regulation, respectively; *i* and *t* are serial numbers of provinces and years, respectively; and *ε* is a random error. The coefficient of each explanatory variable represents the degree of influence of that variable over the explained variable.

### 3.4. Data Sources

The main variables are from EBM and Tobit models. To ensure the completeness and availability of the data on these variables, this study chooses to examine the data about the provinces in China from 2010 to 2018. Note that Hongkong, Macao, Taiwan, and Tibet were excluded because the data on some variables in these provinces were missing for consecutive years. The original data were collected from the statistical yearbooks released by China and its provinces on tourism, energy, transportation, etc. Some missing data were completed through interpolation.

The research data were generated no later than 2018. The data from 2018 to 2021 were not included. The reason is that this paper explores many provinces. The original data on tourism energy input and TCDEE indices of all provinces are not complete after 2018. In some provinces, the relevant data are partly missing in 2019–2021. Thus, the data samples were collected in the time interval of 2010–2018 for data comprehensiveness and availability.

## 4. Results and Discussion

### 4.1. Measured TCDEEs

Based on the proposed index system for TCDEE, the data on various inputs and outputs were entered to MaxDEA. Then, EBM was adopted to measure the provincial TCDEEs in 2010–2018. The results in Table 3 show that China's TCDEEs had obvious provincial differences.

In terms of the mean TCDEE, six provinces, namely, Beijing, Tianjin, Inner Mongolia, Shanghai, Jiangsu, and Guangdong achieved a mean TCDEE of 1 in the sample period. The TCDEEs of these provinces fell on the efficient frontier, reaching the DEA effective state. Geographically, all the six provinces, except for Inner Mongolia, belong to eastern coastal areas. The provinces with high TCDEEs mainly concentrate in eastern coastal areas, thanks to their superior geographical locations, convenient transportation, rich tourism resources, and pursuit of low-carbon tourism. The optimal TCDEE of Inner Mongolia has much to do with its rich tourism resources.

With mean TCDEEs between 0.8 and 0.1, Jilin, Fujian, Liaoning, Heilongjiang, Qinghai, Yunnan, and Zhejiang performed rather well. However, their TCDEEs did not reach the DEA effective state, waiting to be improved. This is because of the redundancy of input production factors: these provinces invest too much manpower, capital, and energy to develop tourism.

Shanxi, Anhui, Hainan, Xinjiang, Guizhou, Shaanxi, Guangxi, Jiangxi, and Hubei ranked in the middle of the country, in terms of the mean TCDEE (0.7–0.8). Located in central and western parts, these provinces witnessed rapid development of tourism in recent years. Nevertheless, the tourism infrastructure in some areas is constructed repeatedly, and little attention is paid to save energy and reduce emissions of tourism. That is why, their TCDEEs were way off the efficient frontier.

The mean TCDEEs of Hunan, Shandong, Ningxia, Henan, Chongqing, Sichuan, Hebei, and Gansu were smaller than 0.7, ranking at the bottom of the country. There is a huge potential for TCDEE improvement in these provinces. Among them, Shandong and Hebei lay in eastern coastal areas. The low TCDEEs of these two provinces are mainly attributable to the redundancy of tourism inputs. Except for Shandong and Hebei, the rest of this group of provinces performed undesirably in the TCDEE. An important reason is the backward transportation and poor infrastructure. In particular, the mean TCDEE of Gansu was merely 0.3029, which is largely associated with the low tourism output.

Overall, different provinces differed significantly in TCDEE. Most eastern provinces had relatively high TCDEEs, while the central and western provinces had relatively low TCDEEs. To promote low-carbon tourism, China must treat central and western parts as the focal points.

Furthermore, China was split into eastern, central, and western parts, according to the geographical location and economic level. The variations of TCDEEs in China and the three parts are displayed in Figure 1.

In the sample period, the TCDEEs in eastern, central, and western parts all changed in the shape of letter N. During 2010–2012, the TCDEEs in China and the three parts exhibited a continuous upward trend. During 2012–2014, the TCDEEs in China and the three parts all declined, and the declining trend lasted to 2016. During 2016–2018, the TCDEEs in China and the three parts were all on the rise.

In addition, there were clear differences in TCDEE between the three parts. In the sample period, the mean TCDEE of the eastern part was as high as 0.8855, which is way above the national average of 0.7979. The mean TCDEE of the central part (0.7788) was close to the national average. The mean TCDEE of the western part (0.7244) fell far behind that of the other two parts. In summary, the TCDEE ranking in China is rather stable in the sample period: eastern part > central part > western part.

### 4.2. Tobit Regression Result

Based on formula (7), TCDEE impactors were estimated by the Tobit model, using Stata 12.0.  Table 4 reports the coefficients of the variables and the significance test results.

The estimation coefficient of the tourism level (TL) was positive but failed the significance test. Thus, the tourism level does not significantly affect TCDEE. The potential reason is as follows: although it brings more economic benefits, a rising tourism level does not truly promote energy conservation and emission reduction in tourism. Currently, the tourism in China is dominated by fashionable tourism. This conventional model of tourism consumes too many energies and discharges lots of pollutants, including carbon dioxide. Therefore, TCDEE improvement hinges on the transformation of fashionable tourism to low-carbon tourism.

Industrial structure (IS) has a prominent negative effect on TCDEE on the level of 1%. This result is closely associated with the internal structure of the tertiary industry in China. At present, the tourism-related sectors account for a large proportion in the tertiary industry, namely, transportation, warehousing, and postal industry; wholesale and retail industry; lodging and catering industry. These sectors consume more energies and emit more carbon dioxide than finance, computer, and software sectors. What is worse, the tertiary industry lacks motivation and vitality, owing to the defects in current institutions and the limited degree-of-freedom for market mechanism. All these issues drag down the TCDEE.

As opposed to our expectation, technical progress (TP) clearly suppresses TCDEE, which is probably due to the direction of technical innovation. Acemoglu et al. [33] divided the technical R&D of enterprises into clean technology and polluting technology. If an enterprise firstly develops polluting technology, then technical innovation only adds to pollutant discharge. In reality, most tourism enterprises seek economic benefits rather than ecological benefits in technical R&D. They prefer polluting technology that takes effect quickly, while creating lots of pollution. Against this backdrop, technical progress can hardly lead to energy conservation and emission reduction unless the government properly guides the R&D direction of enterprises.

Opening-up (OU) has a significant negative correlation with TCDEE. A possible reason is that FDI indeed eases the fund shortage of tourism development. But a lot of funds continue to flow towards the high-pollution tourism sectors. The cash flow pushes up pollutant discharge of tourism and thus lowers TCDEE.

The urbanization level (UL) has a significant positive effect on TCDEE at the level of 1%. This means a high urbanization level is conducive to TCDEE improvement. Every 1% of growth in the urbanization level is followed by 2.697% of increase in TCDEE. As mentioned before, highly urbanized areas tend to have complete infrastructure, possess mature techniques of energy-saving and emission reduction, and make efficient use of resources. Compared with rural residents, urban residents are often well educated and fully aware of the importance of environment. These factors obviously help to promote TCDEE.

Environmental regulation (ES) has an obvious negative impact on TCDEE. This result confirms our hypothesis: if the government investment in environmental pollution control is too high, the resource allocation mechanism of the market would be distorted, which hinders the efficiency improvement. Therefore, the government should not solely rely on mandatory instruments of environmental regulation to better control tourism pollutants but adopt other types of environmental regulation instruments: market incentives, public participation, and voluntary actions.

### 4.3. Discussion

The energy consumption and carbon dioxide emission of tourism grow year by year. As a result, low-carbon economy becomes the optimal choice for Chinese tourism to contribute to global energy conservation and emission reduction [3]. Improving the TCDEE is an important path for tourism to realize sustainable development. Chen et al. [3] claimed that it is reasonable and necessary to decompose the national goal of emission reduction and low-carbon development to different regions in the light of the spatial imbalance of regional economy and tourism development. Focusing on the TCDEE of each Chinese province, this paper discovers a significant provincial difference in TCDEE. Some provinces achieved the optimal TCDEE (efficiency of 1), and some provinces failed to realize the ideal TCDEE. The Chinese provinces had marked a difference in the development of low-carbon economy. Thus, it is necessary to prepare different tourism carbon reduction policies for different provinces. The research results echo with the ideas of Chen et al. [3].

In addition, the distribution of provincial TCDEEs is closely associated with economic growth. In general, the development of tourism economy spurs tourism carbon emission and negatively affects TCDEE. In reality, however, the Chinese provinces pay attention to ecological protection, while promoting tourism economy. This effort drives the low-carbon development of tourism. Taking Heilongjiang as an example, Tang and Huang [34] studied the detachment between carbon dioxide emission and tourism economy growth in 2019 and found that the detachment is basically benign. Thus, they concluded that energy conservation and emission reduction measures have achieved certain effects on promoting the tourism development in Heilongjiang. In this study, the TCDEE of Heilongjiang averaged 0.9007 in the sample period, which is close to the optimal frontier. Therefore, our conclusion that Heilongjiang had a relatively high TCEDD can be strongly supported by Tang and Huang's results [34].

## 5. Conclusions

To realize sustainable development of tourism, the key lies in spurring the saving of energy and emission reduction in the industry. Taking the carbon dioxide emissions of tourism as the undesired output, this study constructs an index system for TCDEE, measures the TCDEEs of 30 provinces in China during 2010–2018, using the EBM model, and analyzes the regional differences of TCDEE. Finally, the TCDEE impactors were tested empirically by the Tobit model.

The previous studies only tackle the TCEDD on the national scale. In this paper, the tourism carbon emission of each Chinese province is measured in the bottom-up manner and used as an undesired output to build a TCEDD index system for comprehensive evaluation. This study not only reduces the research scale of tourism low-carbon development but also compares the TCDEEs between provinces and identifies the factors influencing the provincial difference. These innovative efforts help to formulate scientific policies. The main results are as follows:

1. During the sample period, only six provinces achieved DEA-optimal TCDEEs, namely, Beijing, Tianjin, Inner Mongolia, Shanghai, Jiangsu, and Guangdong. The other provinces failed to reach this state. Besides, there were significant provincial differences in TCDEE. Most provinces with high TCDEEs belong to eastern coastal areas, and those provinces with low TCDEEs concentrate in central and western areas.
2. In the sample period, the TCDEEs in eastern, central, and western parts all changed in the shape of letter N, i.e., the TCDEEs first increased, then declined and eventually rebounded. Furthermore, there were clearly phased variations in regional TCDEEs. In addition, the three parts diverged in terms of TCDEE. The eastern part had the highest TCDEE, followed by the central part, while the western part had the lowest TCDEE. In general, the TCDEE in China gradually decreased from the east to west.
3. According to the Tobit estimation results on TCDEE impactors, TCDEE is significantly enhanced by the urbanization level, greatly inhibited by industrial structure, technical progress, opening-up, and environmental regulation, and not significantly affected by the tourism level.

According to the above conclusions, the following policy suggestions were provided on the low-carbon development of tourism: (1) prepare specific policies on tourism carbon emission reduction for each region; (2) change the traditional fashionable tourism and pay efforts to develop green tourism under the low-carbon economy; (3) accelerate the effective integration of tourism and tertiary industry, optimize the internal structure of the tertiary industry, and reduce the energy consumption intensity of transportation, warehousing, and postal industry, as well as accommodation and catering industries; (4) strengthen the guidance on the direction of technological progress and vigorously promote green innovation; (5) further improve the environmental protection threshold of foreign investment and reduce the entry of foreign-funded enterprises with high pollution and high energy consumption; (6) step up the publicity of environmental protection and enhance people's awareness of environmental protection; (7) give full play to the government in environmental governance and adopt the market-oriented method to control the environmental pollution issues of tourism.

There are still two limitations in this research. Firstly, the tourism carbon emission was estimated. This is a common practice in research when the government has not released the official data of carbon emissions in tourism. However, the estimation may affect the accuracy of the results to a certain extent. Secondly, the sample data were generated between 2010–2018 for the consideration of data availability and comprehensiveness. The short span of the data hinders the long-span analysis of TCDEE and the selection of relevant influencing factors. In the future, the Chinese government is expected to release more data on tourism carbon emission, as it pays more and more attention to carbon neutrality. Then, the authors would carry out deeper analysis on the data released by the government. In addition, the authors would expand the channels of data acquisition. Apart from the statistical yearbooks published by the government, the authors would try to expand the time span of samples by querying relevant data on database websites.

## Figures and Tables

**Figure 1:** Variations of TCDEEs in China and the three parts.

**Table 1:** TCDEE indices.

Variable	Name	Meaning	Unit
Inputs	Labor	Total number of tourism employees in each province	10,000 people
	Capital	Fixed assets in tourism with 2010 as the base year	100 million yuan
	Energy	Tourism energy consumption computed with the tourism consumption stripping coefficient	10,000 tons of standard coal

Outputs	Desired outputs	Total tourism income in each province with 2010 as the base year	100 million yuan
		Number of inbound overnight tourists in each province	10,000 people
	Undesired output	Tourism carbon dioxide emissions estimated by the bottom-up method	10,000 tons

**Table 2:** TCDEE impactors.

Name	Meaning	Unit
Tourism level (TL)	Ln (per capita tourism income)	Yuan/person
Industrial structure (IS)	Tertiary industry output/GDP	%
Technical progress (TP)	R&D expenditure/GDP	%
Opening-up (OU)	Actual utilization of FDI/GDP	%
Urbanization level (UL)	Permanent urban residents/total population	%
Environmental regulation (ES)	Investment on environmental pollution control/GDP	%

**Table 3:** Provincial TCDEEs in 2010–2018.

Province	2010	2011	2012	2013	2014	2015	2016	2017	2018	Mean
Beijing	1.0000	1.0000	1.0000	1.0000	1.0000	1.0000	1.0000	1.0000	1.0000	1.0000
Tianjin	1.0000	1.0000	1.0000	1.0000	1.0000	1.0000	1.0000	1.0000	1.0000	1.0000
Inner Mongolia	1.0000	1.0000	1.0000	1.0000	1.0000	1.0000	1.0000	1.0000	1.0000	1.0000
Shanghai	1.0000	1.0000	1.0000	1.0000	1.0000	1.0000	1.0000	1.0000	1.0000	1.0000
Jiangsu	1.0000	1.0000	1.0000	1.0000	1.0000	1.0000	1.0000	1.0000	1.0000	1.0000
Guangdong	1.0000	1.0000	1.0000	1.0000	1.0000	1.0000	1.0000	1.0000	1.0000	1.0000
Jilin	0.9142	0.9740	1.0000	1.0000	1.0000	1.0000	1.0000	1.0000	1.0000	0.9876
Fujian	0.9833	1.0000	1.0000	0.8273	0.8282	0.8040	0.9278	0.9493	0.9437	0.9182
Liaoning	0.6738	1.0000	1.0000	1.0000	0.6865	0.8823	1.0000	1.0000	1.0000	0.9159
Heilongjiang	0.9312	1.0000	1.0000	0.9231	0.9536	0.8980	0.8619	0.8382	0.7002	0.9007
Qinghai	0.7411	0.7955	1.0000	1.0000	0.6946	0.7840	1.0000	1.0000	1.0000	0.8906
Yunnan	0.8633	0.9223	0.9360	0.7151	0.7078	0.8873	0.8457	0.8670	1.0000	0.8605
Zhejiang	0.9773	0.9406	0.9486	0.7523	0.7508	0.7718	0.7952	0.8318	0.8249	0.8437
Shanxi	0.8101	0.8942	0.9122	0.6096	0.6274	0.7116	0.6335	1.0000	1.0000	0.7998
Anhui	0.8643	0.7765	0.7647	0.8361	0.7070	0.6556	0.6573	0.7384	0.9824	0.7758
Hainan	0.7743	0.8576	0.8406	0.7448	0.6988	0.6795	0.6838	0.7919	0.8630	0.7705
Xinjiang	0.8178	0.8339	0.8029	0.7645	0.7568	0.6718	0.6730	0.7412	0.7473	0.7566
Guizhou	0.6677	0.8358	0.8766	1.0000	0.8374	0.7306	1.0000	0.3864	0.4229	0.7508
Shaanxi	0.6781	0.7273	0.7838	0.7197	0.6858	0.7010	0.7132	0.7650	0.8814	0.7395
Guangxi	0.6644	0.7202	0.7349	0.7515	0.7058	0.6931	0.7509	0.7395	0.7805	0.7267
Jiangxi	0.7969	0.7871	0.8254	0.7569	0.6504	0.6285	0.6286	0.6496	0.6502	0.7082
Hubei	0.6351	0.6832	0.7131	0.8056	0.6741	0.6714	0.6830	0.6928	0.7927	0.7057
Hunan	0.7018	0.6934	0.7242	0.6892	0.6648	0.6383	0.6330	0.7083	0.8075	0.6956
Shandong	0.6424	0.6508	0.6690	0.7330	0.7407	0.7436	0.7108	0.7095	0.6081	0.6898
Ningxia	0.5390	0.6322	0.6773	0.5514	0.6098	0.6571	0.7321	0.7661	0.8762	0.6712
Henan	0.7015	0.7255	0.7271	0.8010	0.7539	0.7463	0.4989	0.4626	0.4871	0.6560
Chongqing	0.6568	0.6891	0.7009	0.5933	0.6031	0.5990	0.6230	0.6306	0.7527	0.6498
Sichuan	0.4833	0.6360	0.6763	0.7394	0.6628	0.5899	0.6507	0.5501	0.5873	0.6195
Hebei	0.7157	0.7179	0.7500	0.6047	0.5485	0.5279	0.5056	0.4791	0.5754	0.6028
Gansu	0.4107	0.4363	0.4115	0.3632	0.1929	0.1871	0.2255	0.2313	0.2680	0.3029

**Table 4:** Regression results of the Tobit model.

Variable	Coefficient	*T*-statistic	*p* value
TL	0.0212	0.87	0.386
IS	−0.9500^*∗∗∗*^	−4.25	≤0.001
TP	−0.0523^*∗∗∗*^	−5.56	≤0.001
OU	−2.1830^*∗∗*^	−2.42	0.016
UL	2.2697^*∗∗∗*^	11.45	≤0.001
ES	−12.8019^*∗∗∗*^	−3.00	0.003
L-likelihood	13.5581		

Note: ^*∗*^, ^*∗∗*^, and ^*∗∗∗*^ are the significance levels of 10%, 5%, and 1%, respectively.

## Data Availability

The data used to support the findings of this study are available from the corresponding author upon request.

## References

[1] Becken S. (2007). Tourists’ perception of international air travel’s impact on the global climate and potential climate change policies. *Journal of Sustainable Tourism*.

[2] Gössling S. (2002). Global environmental consequences of tourism. *Global Environmental Change*.

[3] Chen L., Thapa B., Yan W. (2018). The relationship between tourism, carbon dioxide emissions, and economic growth in the Yangtze River Delta, China. *Sustainability*.

[4] Wu P., Shi P. (2011). An estimation of energy consumption and CO_2_ emissions in tourism sector of China. *Journal of Geographical Sciences*.

[5] Sun Y. Y. (2016). Decomposition of tourism greenhouse gas emissions: revealing the dynamics between tourism economic growth, technological efficiency, and carbon emissions. *Tourism Management*.

[6] Scott D., Peeters P., Gössling S. (2010). Can tourism deliver its “aspirational” greenhouse gas emission reduction targets. *Journal of Sustainable Tourism*.

[7] Peeters P., Dubois G. (2010). Tourism travel under climate change mitigation constraints. *Journal of Transport Geography*.

[8] Perch-Nielsen S., Sesartic A., Stucki M. (2010). The greenhouse gas intensity of the tourism sector: the case of Switzerland. *Environmental Science & Policy*.

[9] Berners-Lee M., Howard D. C., Moss J., Kaivanto K., Scott W. (2011). Greenhouse gas footprinting for small businesses-the use of input-output data. *The Science of the Total Environment*.

[10] Gössling S., Peeters P., Ceron J. P., Dubois G., Patterson T., Richardson R. B. (2005). The eco-efficiency of tourism. *Ecological Economics*.

[11] Mayor K., Tol R. S. J. (2010). Scenarios of carbon dioxide emissions from aviation. *Global Environmental Change*.

[12] Amado C. A. F., Santos S. P., Serra J. M. M. (2017). Does partial privatisation improve performance? Evidence from a chain of hotels in Portugal. *Journal of Business Research*.

[13] Kularatne T., Wilson C., Månsson J., Hoang V., Lee B. (2019). Do environmentally sustainable practices make hotels more efficient? a study of major hotels in Sri Lanka. *Tourism Management*.

[14] Barros C. P., Matias Á. (2006). Assessing the efficiency of travel agencies with a stochastic cost Frontier: a Portuguese case study. *International Journal of Tourism Research*.

[15] Fuentes R., Alvarez-Suarez A. (2012). Productivity of travel agencies in Spain: the case of Alicante. *Service Industries Journal*.

[16] Sarkis J., Talluri S. (2004). Performance based clustering for bench marking of US airports. *Transportation Research Part A: Policy and Practice*.

[17] Ladino M. D. M., Buitrago D. M. B. (2022). Proposal for a mining-touristic route in parque minero industrial Mochuelo Bajo, Bogota. A look from the environmental, social and productive factor. *International Journal of Sustainable Development and Planning*.

[18] Kytzia S., Walz A., Wegmann M. (2011). How can tourism use land more efficiently? a model-based approach to land-use efficiency for tourist destinations. *Tourism Management*.

[19] Zhang T., Chi Y. Y. (2020). Evaluation of green economic development abilities of Hubei Province in 2008–2018. *International Journal of Sustainable Development and Planning*.

[20] Charnes A., Cooper W. W., Rhodes E. (1978). Measuring the efficiency of decision making units. *European Journal of Operational Research*.

[21] Banker R. D., Charnes A., Cooper W. W. (1984). Some models for estimating technical and scale inefficiencies in data envelopment analysis. *Management Science*.

[22] Zhou P., Ang B. W., Wang H. (2012). Energy and CO_2_ emission performance in electricity generation: a non-radial directional distance function approach. *European Journal of Operational Research*.

[23] Tone K. (2001). A slacks-based measure of efficiency in data envelopment analysis. *European Journal of Operational Research*.

[24] Tone K., Tsutsui M. (2010). An epsilon-based measure of efficiency in DEA: a third pole of technical efficiency. *European Journal of Operational Research*.

[25] Zha J., Yuan W., Dai J., Tan T., He L. (2020). Eco-efficiency, eco-productivity and tourism growth in China: a non-convex metafrontier DEA-based decomposition model. *Journal of Sustainable Tourism*.

[26] Becken S., Simmons D. G., Frampton C. (2003). Energy use associated with different travel choices. *Tourism Management*.

[27] Becken S., Patterson M. (2006). Measuring national carbon dioxide emissions from tourism as a key step towards achieving sustainable tourism. *Journal of Sustainable Tourism*.

[28] Lin T. P. (2010). Carbon dioxide emissions from transport in Taiwan’s national parks. *Tourism Management*.

[29] Sun Y., Hou G., Huang Z., Zhong Y. (2020). Spatial-temporal differences and influencing factors of tourism eco-efficiency in China’s three major urban agglomerations based on the super-EBM model. *Sustainability*.

[30] Qiu X., Fang Y., Yang X., Zhu F. (2017). Tourism eco-efficiency measurement, characteristics, and its influence factors in China. *Sustainability*.

[31] Sinn H. W. (2008). Public policies against global warming: a supply side approach. *International Tax and Public Finance*.

[32] Tobin J. (1958). Estimation of relationships for limited dependent-variables. *Econometrica*.

[33] Acemoglu D., Aghion P., Bursztyn L., Hemous D. (2012). The environment and directed technical change. *The American Economic Review*.

[34] Tang Z., Huang T. Y. (2021). Carbon dioxide emission measurement and its spatiotemporal evolution of tourism industry in Heilongjiang province, China. *Advances in Meteorology*.

